The article "A Case Presentation Based on Incidental Diagnosis of Atrial Myxoma in a Patient Presenting With Atrial Fibrillation and Suspected Carney Complex" was published in 2022. Journal: Cureus.

# A Case Presentation Based on Incidental Diagnosis of Atrial Myxoma in a Patient Presenting With Atrial Fibrillation and Suspected Carney Complex

**DOI:** 10.7759/cureus.21157

**Published:** 2022-01-12

**Authors:** Zahid Khan, Umesh Kumar Pabani, Animesh Gupta, Sunaina Lohano, Gideon Mlawa

**Affiliations:** 1 Cardiology, Royal Free Hospital, London, GBR; 2 Internal Medicine, Barking, Havering and Redbridge University Hospitals National Health Services Trust, London, GBR; 3 Acute Internal Medicine, Barking, Havering and Redbridge University Hospitals National Health Services Trust, London, GBR; 4 Geriatrics, Newham University Hospital, London, GBR; 5 Internal Medicine and Diabetes and Endocrinology, Barking, Havering and Redbridge University Hospitals National Health Services Trust, London, GBR

**Keywords:** therapeutic anticoagulation, atrial fibrillation recurrence, acromegaly and diabetes, diabetic retinopathy, diabetic nephropathy (dn), diabetes mellitus type 2, carney complex, atrial myxoma

## Abstract

We present the case of a 54-year-old lady who presented to hospital with palpitations and was diagnosed with atrial fibrillation with rapid ventricular response. She was given intravenous metoprolol 5 mg initially followed by a further 5 mg and was commenced on bisoprolol 2.5 mg once daily. She reverted back to normal sinus rhythm and was referred for echocardiography following an episode of paroxysmal atrial fibrillation. The echocardiogram showed a large mobile atrial myxoma in the left atrium and mild-to-moderate mitral regurgitation with preserved left ventricular function. Her past medical history includes transsphenoidal surgery for acromegaly in 1979, followed by radiotherapy and partial thyroidectomy for goitre. Her chest radiograph was normal and blood results were unremarkable. She was accepted for inpatient transfer to a cardiothoracic centre for surgical removal of atrial myxoma. She underwent surgery with successful excision of the atrial myxoma, and biopsies confirmed the mass to be atrial myxoma. The surgery was complicated by the patient developing atrial fibrillation with fast ventricular response that was chemically cardioverted with an intravenous loading dose of amiodarone 300 mg over 2 hours followed by 900 mg infusion over 24 hours. She had follow-up in the outpatient clinic with cardiology and endocrine specialists for a year and no recurrence of myxoma was noted. Her blood tests including growth hormone and thyroid function tests were normal.

## Introduction

Carney complex (CNC) is an autosomal genetic syndrome characterized by spotty pigmentation of the skin, endocrinopathy, and endocrine and nonendocrine tumours such as myxomas of the skin, heart, breast, and other sites [1]. The CNC is a rare disease and about 750 cases have been reported worldwide so far. The exact prevalence of the condition is unknown, and it is characterized by multiple neoplasms that may include neuroendocrine and cardiac tumours [1]. The majority of cardiac myxomas show sporadic appearance and less than 10% show a family inheritance pattern [2]. The most common cardiac site involved is left atria and it accounts for 75-80% of the total cardiac myxoma reported followed by the right atrium. About 50% of cardiac myxomas have bilateral origin [3]. The common cause of death in a patient with CNC is cardiac cause or due to complications from the cardiac myxoma such as embolic stroke, cardiomyopathy, or arrhythmia. Therefore, difficult diagnostic decision must be made in patients with atrial myxoma and suspected CNC and regular follow-up are required to prevent sudden cardiac death and embolic events in these patients. Reports of biatrial myxoma are rare, but it is not unheard of, although in most cases, a single myxoma reaches both atria. It is important to investigate patients with multiple endocrine tumours for CNC and an echocardiography should be performed in these patients to assess for the presence of atrial myxoma.

The article "A Case Presentation Based on Incidental Diagnosis of Atrial Myxoma in a Patient Presenting With Atrial Fibrillation and Suspected Carney Complex" was published in 2022. Journal: Cureus.

## Case presentation

We present the case of a 54-year-old female who presented to the emergency department (ED) with atrial fibrillation (AF) with rapid ventricular response. Her only past medical history consists of transsphenoidal surgery for acromegaly in 1979, followed by radiotherapy and partial thyroidectomy for goitre. She did not have any echocardiogram prior to the radiotherapy or surgery according to the patient although we could not access any of her previous records as the patient was registered with a different general practitioner at that time. However, she had two echocardiograms in 2008 and 2009 and they were reported as normal. Her regular medications include cabergoline 250 mcg once weekly, hydrocortisone 15 mg in the morning, 5 mg mid day and 5 mg in the evening, levothyroxine 125 mcg once daily, and bisoprolol 5 mg once daily.

In the ED, she was initially rate controlled with metoprolol, followed by an increased dose of bisoprolol 7.5 mg once daily regularly. She had inpatient echocardiogram once her heart settled down below 100 beats per minute and she reverted to normal sinus rhythm. She was commenced on rivaroxaban 20 mg once daily in view of her CHADSVASC score =2. The echocardiogram showed normal left ventricular ejection fraction >60%, mild left atrial dilatation, and a large left atrial mobile mass (5.6 cm × 3.0 cm in diameter), which was homogeneous and regular in appearance, adhered to the interatrial septum with no gradient of stenosis or signs of regurgitation (Figures 1, 2, 3).

The article "A Case Presentation Based on Incidental Diagnosis of Atrial Myxoma in a Patient Presenting With Atrial Fibrillation and Suspected Carney Complex" was published in 2022. Journal: Cureus.

**Figure 1:** Echocardiography parasternal long-axis view showing left atrial myxoma

**Figure 2:** Echocardiography apical four-chamber view showing left atrial myxoma

**Figure 3:** Echocardiography parasternal short-axis view showing left atrial myxoma

On physical examination, she had pigmented freckles, coarse facial features, and big hands suggestive of acromegaly. She was transferred to a cardiothoracic centre for surgical resection of the left atrial myxoma after a week of inpatient admission. Her surgery was complicated by development of AF with fast ventricular response, and she had chemical cardioversion with amiodarone. She stayed in the hospital for seven days and was discharged home.

She represented to the hospital two months later with shortness of breath and associated chest pain. She had raised inflammatory markers as shown in Table 1 and the chest X-ray showed right-sided consolidation. Her electrocardiogram showed normal sinus rhythm and she had normal troponin level.

**Table 1:** Table showing laboratory investigations result of the patient

Blood Test	Value	Normal Value
Haemoglobin	134	133-173 g/L
White cell count	20	3.8-11 × 10^9^/L
Neutrophil	15	2-7.5 × 10^9^/L
C-reactive protein	88	0-5 mg/L
Urea	7.0	2.5-7.8 mmol/L
Creatinine	82	59-104 μmol
Sodium	138	133-146 mmol/L
Potassium	4.5	3.5-5.3 mmol/L
Growth hormone level	0.39 ng/mL	<10 ng/mL
T4	11.5	5-12 μg/dL

She had outpatient cardiology follow-up in six months' time and repeat echocardiography did not show any recurrence of myxoma. The patient remains stable with no evidence of growth hormone excess, and a growth hormone level of 0.39 mcg/L, T4 17.5, and normal cortisol day curve as shown in Table 1. Her last magnetic resonance imaging (MRI) pituitary showed resolution of the pituitary adenoma (minimal amount of pituitary gland tissue in the pituitary fossa). She remained stable on 25 mg of split-dose hydrocortisone when she was seen in the endocrine outpatient clinic.

## Discussion

This patient was diagnosed with acromegaly in 1979 and CNC was first described in 1985 by J. Aiden Carney and he described the key clinical manifestation to be spotty pigmentation, endocrine overactivity, and myxoma [4]. The two common mutations considered to be responsible for the disease include the PRKAR1A gene on chromosome 17q22-24 and another gene called CNC2 on chromosome 2p16 [5,6].

Although the exact prevalence is unknown, and the diagnosis is often delayed owing to its rarity and complexity, patients with some rare non-endocrine tumours, such as cardiac myxomas and osteochondromyxomas, should be investigated for CNC [7,8]. The most common manifestation of CNC includes lentigines and blue nevi followed by cardiac myxomas, which are notorious for recurrence and do not show any age, sex, or location preponderance [9,10].

The article "A Case Presentation Based on Incidental Diagnosis of Atrial Myxoma in a Patient Presenting With Atrial Fibrillation and Suspected Carney Complex" was published in 2022. Journal: Cureus.

In another case report, a 47-year-old male patient presented with a one-year history of exertional dyspnoea and palpitation, admitted with complaints of syncopal attacks of sudden onset and a car bike accident four years ago. His X-rays of the right lower limb at that time showed lytic lesion in the distal end of the right femur with destruction of the lateral cortex and a pathological fracture and periosteal reaction along the lateral aspect of distal femur. Histological findings from the biopsy were supportive of the diagnosis of giant cell tumour of the bone. He also had multiple spotty pigments on his trunks and was diagnosed with superficial angiomyxoma. Echocardiogram showed left atrial myxoma with moderate mitral stenosis, and coronary angiography was normal in this patient and had successful removal of the left atrial myxoma [9]. The patient in our case also had acromegaly, skin pigmentation, and atrial myxoma and this confirms the findings from previous studies that these patients tend to have cardiac and non-cardiac tumours. The patient in our case was diagnosed with acromegaly in 1979 and CNC was first discovered in 1985, which is the likely explanation for her being misdiagnosed.

When CNC was discovered by J Carney in 1985, there were approximately 150 patients affected by the disease worldwide, and the common organs involved by myxoma included the heart, skin, and breast. The common skin sites for myxoma are eyelids, external ear canal, and nipples and recurrence is quite common after excision of the primary lesion. The lentigines typically involve the centrofacial area, including the vermilion border of the lips, and the conjunctiva, especially the lacrimal caruncle and the conjunctival semilunar fold. On the other hand, the blue nevi occur on the face, trunk, and limbs, but sparing hands and feet [10].

Endocrine problems arising from CNC include Cushing's syndrome, acromegaly, and sexual precocity. The schwannomas most commonly affect the upper gastrointestinal tract and sympathetic nerve chains, but a few have occurred in the skin [10,11].

Atrial myxoma can also run in families and Wang L, et al. (2018) presented a case report based on three family members who had atrial myxoma. The first family member to be diagnosed with the condition had recurrent atrial myxoma and had surgical resection twice, and on screening of the other family members, two more family members were also found to have atrial myxoma associated with CNC [11]. The exact prevalence of the disease in Asian families is not known and both the brother of the proband and nephew of the proband were confirmed with the diagnosis of atrial myxoma and underwent surgical resection. The nephew just like the proband underwent surgical resections twice for atrial myxoma. It is also important to mention that the father of the proband had sudden cardiac death at an age of 43 without a proper diagnosis [11]. 

The article "A Case Presentation Based on Incidental Diagnosis of Atrial Myxoma in a Patient Presenting With Atrial Fibrillation and Suspected Carney Complex" was published in 2022. Journal: Cureus.

It is important to follow up these patients regularly. The current guidelines based on the advice from previous studies suggest that these patients should have follow-up arrangement as shown in Table 2.

**Table 2:** Follow-up recommendations for patients with Carney complex and atrial myxoma

Follow-up recommendations for patients with Carney complex and atrial myxoma
1. Annual echocardiogram from childhood, and if the patient was diagnosed with atrial myxoma once, they should have echocardiogram twice a year [12].
2. These patients need regular skin evaluations.
3. Regular bloods tests including levels of growth hormone, prolactin, and insulin-like growth factor 1 beginning in adolescence, urinary free cortisol, and screening for Cushing's syndrome.
4. Thyroid gland (neck) clinical examinations and with ultrasound, if needed.
5. Computerized tomography scan of adrenal glands for the detection of primary pigmented nodular adrenocortical disease; pituitary MRI, and MRI of brain, spine, chest, abdomen, retroperitoneum, and pelvis for the detection of psammomatous melanotic schwannomas [12,13].
6. Ultrasound testicles annually for the detection and follow-up of large cell-calcifying Sertoli cell tumours in men.
7. Transabdominal ultrasound of the ovaries in women.

The average life span of patients with CNC is 50-55 years based on the current data; however, this can be normal based on careful surveillance as the most common cause of death in these patients is due to complications arising from heart myxomas, such as embolic cardiovascular or cerebrovascular events, post-operative cardiomyopathy and cardiac arrhythmia, and metastatic psammomatous melanotic schwannomas and other cancer-related complications [13,14].

## Conclusions

Arriving at a unifying diagnosis can be difficult and is often delayed as demonstrated in this case report. Patients with CNC should have an annual symptom review as well as blood tests for insulin-like growth factor 1, prolactin, and thyroid function. They also need to have annual echocardiogram as well as pituitary MRI, thyroid, and testicular/ovarian ultrasound. Annual colonoscopy is recommended if acromegaly is part of CNC.

Our patient's record shows that she had echocardiogram in 2008 and 2010 and there was no mention of atrial abnormality. This case report highlights the importance of annual echocardiography in patients with CNC or twice-yearly echocardiography in patients with recurrent atrial myxomas. Additionally, family members of the patients with CNC should also be screened for atrial myxomas.
